The article "Qing Zao Fang (QZF) Alleviates the Inflammatory Microenvironment of the Submandibular Gland in Sjögren's Syndrome Based on the PI3K/Akt/HIF-1α/VEGF Signaling Pathway" was retracted in 2023. Reasons: signs of a paper mill; suspected computer-generated content; unreliable results or conclusions; lack of ethics approval or compliance.

# Qing Zao Fang (QZF) Alleviates the Inflammatory Microenvironment of the Submandibular Gland in Sjögren's Syndrome Based on the PI3K/Akt/HIF-1*α*/VEGF Signaling Pathway

**DOI:** 10.1155/2022/6153459

**Published:** 2022-01-31

**Authors:** Ping Zeng, Wei Liu, Xiaochun Yang, Shumin Zhang, Shaopeng Du, Yihua Fan, Longmei Zhao, Aihua Wang

**Affiliations:** ^1^First Teaching Hospital of Tianjin University of Traditional Chinese Medicine, Tianjin 300193, China; ^2^National Clinical Research Center for Chinese Medicine Acupuncture and Moxibustion, Tianjin, 300381, China; ^3^Tianjin University of Traditional Chinese Medicine, Tianjin 301617, China; ^4^Guizhou University of Traditional Chinese Medicine, Guiyang 550025, China

## Abstract

Sjögren's syndrome (SS) which could lead to a disorder of our immune system is a chronic autoimmune disease characterized by invading exocrine glands such as salivary glands and lacrimal glands and other exocrine glands. Its common symptom is dry mouth and dry eyes, often accompanied by a large number of lymphocyte infiltrations and can involve other organs to cause complex clinical manifestations. In this study, we aimed at investigating the effect of QZF in SS, identifying the molecular mechanism in modulating autoimmune response, and determining the important roles of these factors' function as a modulator in the pathogenesis of SS. The NOD mice were utilized to establish the rats' model of Sjögren's syndrome. After 10 weeks' hydroxychloroquine and QZF in different dose interference, submandibular gland tissue was collected. The therapeutic effect of QZF on SS rats was identified, and the results suggest the comparable potential to hydroxychloroquine. In submandibular gland tissue, interleukin- (IL-) 17 was significantly lower in high-dose QZF than that in SS rats and the focal lymphocytes were highly attenuated. Moreover, we found that PI3K/Akt signals were activated and the downstream HIF-1*α*/VEGF signals were enhanced in SS rats whose protein expression could be inhibited by QZF treatment. In addition, QZF could modulate autophagy in submandibular gland tissue and then inhibit the inflammation response and therefore facilitate the tissue repair.

## 1. Introduction

Sjögren's syndrome (SS) could lead to a disorder of our immune system by invading exocrine glands causing lymphocyte infiltration and thus disturbing immune response in salivary and lacrimal glands. It is a chronic autoimmune disease with autoimmune system disorder in salivary and lacrimal glands represented as two main symptoms in patients (dry mouth and dry eyes) [1, 2]. The disease has affected approximately 1% of the general population among all ages, and up to 3% of people over the age of fifty, with women accounting for more than 90% of diagnosed cases [3]. Different from the secondary Sjogren's syndrome which is suffered on the basis of other autoimmune disorders like rheumatoid arthritis (RA) and systemic lupus erythematosus (SLE), the primary Sjögren's syndrome is encountered alone [4]. Systemic manifestations occurred in 30-40 percent of patients with pSS and cause an adverse effect on patients in quality of life. Furthermore, the fatality rate was increased year by year among the patients with pSS [5]. Thus, an effective strategy for the treatment of SS is imperatively and urgently needed.

Interleukin- (IL-) 17A was discovered in 1995 and for the first time reported in 2000 to have a great correlation with inflammation and infection [6, 7]. The T help type 17 (Th17) cells have been reported in 2005 as another subgroup of CD4+ T cells which could secrete IL-17 [8]. At the same time, some studies have shown that the onset of SS is related to the differentiation of T cell subsets and is intimately correlated to the expression of the proinflammatory factor IL-17 in recent years [9, 10]. IL-17A is a powerful proinflammatory factor that can be vastly secreted by Th17 cells; moreover, IL-17A also can act on a variety of cell types for the inducing expression of cytokines including proinflammatory cytokines, chemokines, and matrix metalloproteinases [11, 12]. Similar to Th1 and Th2 cell subgroups, the steroid receptor type nuclear receptor ROR*γ*t also is the corresponding major regulators of Th17 cells [13]. Studies have shown that ROR*γ*t can promote the expression of IL-17A and IL-17F by naive T cells and therefore regulate the secretion of IL-17 [14], while regulatory T (Treg) cells which can inhibit immune response play an important role in immune balance maintaining and regulating immunity [15].

It is found that Th17 and Treg cells play opposite roles in inflammatory and immune response and maintain a dynamic balance [16]. Once Th17/Treg is imbalanced, it may cause the occurrence of autoimmune diseases because of a vast secretion of IL-17 leading to the abnormal immune response of lymphocytes and thus the crucial role of this imbalance in the pathogenesis of SS [17, 18]. Th17 not only participates in the occurrence and development of SS but also has a positive correlation with the status of disease [15–19]. Among them, IL-17A and IL-17F are the most distinctive cytokines in this family. Once the IL-17A and IL-17F are activated, a strong inflammatory response was triggered and then induces the generation of potential proinflammatory cytokines to promote the inflammatory response and the neutrophil proliferation, maturation, and accumulation [20]. IL-17A is also related to the degree of lymphocyte infiltration and clinical indicators in patients with SS. As the degree of lymphocyte infiltration increases, the expression of IL-17A increases. The lymphocyte infiltration degree around the salivary ducts is thus positively relevant to the level of gland damage. The higher the IL-17A mRNA expression is, the more severe the tissue damage [21]. In SS animal experiments, immunization of wild-type C57BL/6 mice with salivary gland protein can induce obvious SS symptoms, accompanied by an increase in cervical lymph node Th17 cells, salivary gland inflammation, and lymphocyte infiltration, while there are no SS symptoms and histopathological changes in IL-17A knockout mice [22].

Hypoxia-inducible factor-1 (HIF-1), a heterodimer composed of HIF-alpha and HIF-beta subunits, is a type of transcriptional active factor related to hypoxic stress found in hypoxia-induced nuclear extracts when Semenza and Wang firstly found and detected the expression of erythropoietin gene in 1992 [23]. The HIF-1 can activate the specific hypoxia susceptibility genes and initiate the transcription of hypoxia response-related elements, thereby regulating the expression of downstream genes of interest and mediating the adaptation of cells to hypoxia reaction [24–26].

The research on the mechanism of statin drugs in tumor treatment by Wang et al. [27] was implemented; the findings were that there are binding sites HRE on the vascular endothelial growth factor (VEGF) gene that can interact with HIF-1 and combine with it to form a transcription initiation complex and initiate the transcription of the corresponding target gene. At the same time, HIF-1*α* also reversely enhances the expression level of the VEGF gene and the stability of its expression products which constitutes positive feedback regulation and continuously promotes the formation of new blood vessels. Studies have found that the expression of HIF-1 in rheumatoid arthritis (RA) patients' rheumatoid arthritis synovial fibroblasts (RASFs) is increased. The HIF-1 may enhance IL-8 and IL-33 expression, mitochondrial membrane potential, and the expression of VEGF in RASFs, thus aggravating inflammation, cartilage destruction, and angiogenesis and participating in the pathogenesis of RA [28, 29]. In addition, studies have reported that HIF-1 can affect the ratio of Th17 and Treg cells' number, thereby causing an immune imbalance and ultimately inducing the onset of systemic lupus erythematosus (SLE) [30]. Shah et al. [31]. found that the expression of salivary gland autophagy-related genes was elevated in patients, while the mammalian target of rapamycin (mTOR) as a protein that mediates the function of antigen-presenting cells and autophagy, the expression inhibition of mTOR can decrease autophagy-related and inflammation-related genes and induce autophagy recovery. Therefore, we believe that modulating autophagy activity and inhibiting angiogenesis may become a fresh direction for the treatment strategy of autoimmune diseases in the future.

In recent years, the researches on hypoxia mediated by HIF-1 are receiving attention from academia. HIF-1 is widely involved in many cell signaling pathways correlated with oxygen perception and response and is identified as the transduction center of hypoxia signals regulating [32]. It was found in several studies that HIF-1 can impact the immune imbalance of Th17/Treg cells through mediating the Th17/Treg cell expression, thereby causing the occurrence of autoimmune diseases [33]. Phosphatidylinositol-3 kinase (PI3K) can be activated under hypoxia and bind to downstream protein kinase B (Akt) to phosphorylate Akt. The phosphorylated Akt can enhance the activity of HIF-1*α*, thus initiating the transcription of HIF-1-related target genes and ultimately accelerating cell proliferation and suppressing cell apoptosis [34–36]. Therefore, in-depth research on the molecular mechanism of the PI3K/Akt/HIF-1*α* signaling pathway regulating Th17 in the pathogenesis and maintenance of SS is hypothesized to put forward new ideas for the medical treatment of SS.

In our study, we aimed to examine the traditional Chinese medicine QZF effect on pSS and explore the mechanism of it. Initially, the SS mouse model was established; QZF was given to the model mouse to investigate the therapeutic effect on alleviating SS. Multiple methods were implemented, the therapeutic effect of QZF on SS was identified, and further PI3K/Akt/HIF-1*α*/VEGF signaling pathway participation was studied and discussed. It is hypothesized that Sjögren's syndrome could be alleviated by QZF based on the PI3K/Akt/HIF-1*α*/VEGF signaling pathway. Our data demonstrate the efficacy of QZF on alleviating the inflammation, modulating autophagy of the submandibular gland in SS rats by inhibiting PI3k/Akt/HIF-1*α*/VEGF signaling pathways. It is expected to provide an insight into the clinical applications using pharmacological analysis for the treatment of SS.

## 2. Materials and Methods

### 2.1. Sjögren's Syndrome Model Establishment and Administration

The animal experiments comply with the ethical standards, and the experimental protocol was approved by the Second Affiliated Hospital of Guizhou University of Chinese Medicine (KY2019012/20190107). The spontaneous SS model in NOD mice was used for experimental study. A total of 75 SPF female NOD mice and 15 SPF female NOD mice aged 8 weeks were prepared for animal experiment. The SS animals were induced as described previously by Lin et al. [22]. All animals were obtained from Beijing Vital River Laboratory Animal Technology Co., Ltd. (Beijing, China). 15 NOD mice were used for the blank control group. Five groups (15 each) were randomly separated from NOD mice: SS, SS+HCQ-treated, SS+low-dose QZF-treated, SS+medium-dose QZF-treated, and SS+high-dose QZF-treated groups. The prescription of QZF is supplied by the pharmacy of the Second Affiliated Hospital of Guizhou University of Chinese Medicine. The animals of the QZF-treated group were administered by QZF in terms of the animal body weights; low-dose QZF water decoction (14.5 g·kg^−1^/d), medium dose (29 g·kg^−1^/d), and high dose (58 g·kg^−1^/d) were given orally once a day, respectively [37, 38]. The positive control group was given hydroxychloroquine (40 mg·kg^−1^/d) water solution for consecutive 10 weeks, while an equal amount of normal saline (0.2 mL/d) was administered by gavage to the negative control group Sjögren's syndrome model and the control group. Finally, after ten weeks of continuous administration, the mice were sacrificed by severed neck; the bilateral submandibular gland tissues were quickly removed and stored or treated for later use.

### 2.2. Western Blot

The ultrasonic cell crusher (SM-650A, SHUNMATECH) was used for submandibular gland tissue protein extraction, the prepared minced tissue was placed in it for cell disruption and then centrifuged for cell debris, and the whole protein was extracted. The experiment begun with SDS-PAGE electrophoresis for separating proteins of different molecular weights. Then, proteins were transferred to polyvinylidene fluoride (PVDF) membranes, washed with TBST for 1 min, and blocked with phosphate-buffered saline (PBS) containing 5% blotting grade for 1 h. Followed by blocking, three times washing each for 5 min was performed with Tris-buffered saline with Tween 20 (TBST). The appropriate primary antibody (1 : 1000) incubation was performed on transferred membrane at 4°C overnight and then followed by 1 h IgG (1 : 2000, ABclonal) incubation at room temperature. The protein band imaging was performed by the enhanced chemiluminescence (ECL) system following the manufacturer's instructions. The catalogue number and brand of used primary antibodies were listed in the following: anti-PI3K (4228T, ABclonal), anti-p-PI3K (4228T, CST), anti-AKT (A17909, ABclonal), anti-p-AKT (4060T, ABclonal), anti-HIF-1*α* (A16873, ABclonal), anti-VEGF (A12303, ABclonal), anti-IL-17A (A0688, ABclonal), anti-LC3 I/II (A19665, ABclonal), and *β*-actin (1 : 2000, AC026, ABclonal).

### 2.3. mRNA Quantification Using Quantitative Real-Time PCR

In light of the manufacturer's instructions, total RNA was extracted with the RNAiso Plus reagent (Takara). The Goldenstar™ RT6 cDNA Synthesis Kit was employed for reverse transcription synthesis of cDNA (Beijing Qingke Biotechnology Co., Ltd.) as per the manufacturer's instructions of use. The 7500 Real-Time PCR System (Thermo Fisher Scientific, Inc.) was used for real-time PCR analyses with 2x T5 Fast qPCR Mix (SYBR Green I) (Beijing Qingke Biotechnology Co., Ltd.). The corresponding primers applied in RT-qPCR are listed in Table 1. The reaction system was as follows: 95°C for 30 sec, followed by 40 cycles of 95°C for 5 sec, 55°C for 30 sec, and 72°C for 30 sec. *β*-Actin was then utilized as an internal control and repeated 3 times for each sample. All procedures were performed in triplicate.

### 2.4. Histopathology

The submandibular gland tissue was initially fixed with 4% paraformaldehyde (Solarbio, Shanghai, China) in PBS at 4°C for 24 h for subsequent pathology analysis and then cut into 3-microm-thick sections after embedding in paraffin. Sections were deparaffinized, and the hematoxylin (Jiancheng, Nanjing, China) and eosin (Jiancheng, Nanjing, China) (H&E) were used for tissue staining. Stained tissues' images were observed using a light microscope (Olympus FSX100; Olympus Corporation).

### 2.5. Immunohistochemistry

Immunohistochemistry (IHC) analysis was carried out by using MaxVisionTM techniques (Maixin Bio, China) based on the manufacturer's instructions. Firstly, the submandibular gland tissue was fixed for preventing from falling off the slide and easy to store, 4% paraformaldehyde (Solarbio, Shanghai, China) was generally used for fixation and then dehydrated and paraffin-embedded, and 5 *μ*m slides were sectioned. The deparaffinization and hydration were performed on the tissue sections; the slides were then incubated with 3% H_2_O_2_ (Sinopharm, China) for 10 min and 0.1% trypsin (Beyotime, China) for 20 min. The specified primary antibodies were incubated at 4°C overnight for antigen detection and then incubated with HRP-polymer-conjugated secondary antibody at 37°C for 1 hour. The slides were then stained by using chromogenic reagent diaminobenzidine (DAB, Zhongshan, Beijing, China) for 3 min and counterstained with hematoxylin (Jiancheng, Nanjing, China). An inverted microscope (Olympus, Japan) was employed for image acquisition. The primary antibodies anti-IL-6 (ab208113), anti-IL-10 (ab189392), and anti-IL-17 (ab79056) were purchased from Abcam (Cambridge, UK).

### 2.6. TUNEL Assay

A TUNEL Kit (cat. no. 11684817910; Roche Diagnostics (Shanghai) Co., Ltd.) was used according to manufacturer guidelines to detect apoptosis following three cycles of washing with PBS. Briefly, the submandibular gland tissue slides were permeabilized with 0.1% Triton X-100, followed by fluorescein isothiocyanate- (FITC-) labeled UTP (deoxyuridine triphosphate) staining for 1 h at 37°C. The sections of submandibular gland tissue cells were stained. Imaging was performed using a light microscope (Olympus FSX100; Olympus Corporation) at magnification ×400 folds.

### 2.7. Statistical Analyses

All analyses were conducted by using GraphPad Prism version 9.0 (GraphPad Software; San Diego CA). One-way analysis of variance (ANOVA) with Tukey post hoc testing was applied to detect statistical significance among three or more groups, and *P* < 0.05 was considered significant. Data are presented as mean ± standard error (SD).

## 3. Results

### 3.1. QZF Could Attenuate Pathogenesis of Sjögren's Syndrome in the SS Model

Several methods were adopted to explore the therapeutic effect of QZF on Sjögren's syndrome rats. Dry mouth and dry eyes due to the impaired function of salivary and lacrimal glands are some of the clinical symptoms of Sjögren's syndrome. After two weeks of adaptive feeding in eight weeks aged rats, the weekly water intake of each group of rats was recorded from the eleventh week. In contrast to the control group, the average water intake of mice in the model group was significantly increased, and the water intake preferred an increasing trend with the development of the disease; compared with the SS model, mice in the high- and medium-dose QZF group and the hydroxychloroquine group indicate decreased average water intake at 16 weeks of age and the water intake showed a continuous decreasing trend as the course of the disease progressed (Figure 1(a)). The submandibular gland index in the SS model decreased than that in the control group (*P* < 0.001). The submandibular gland index of the hydroxychloroquine group and high dose of QZF increased in comparison with the SS model (*P* < 0.001) (Figure 1(b)). Comparative curative effects were observed in hydroxychloroquine and high-dose QZF without significant difference in index.

The submandibular gland tissues of different groups were sectioned, and HE stained to observe the tissue morphology, and the results are exhibited in Figure 1(c). As is shown, the acinus of the submandibular gland tissue is homogeneous in size and tightly arranged in the control group. Compared with the control group, focal infiltration of lymphocytes was found, and acinar cells are significantly reduced, ducts are dilated and fused, and some tissues are degenerated and necrotic in the SS group. The hydroxychloroquine group shows a small amount of lymphocyte infiltration, some ducts were dilated, and acinar cells were reduced compared with the control group. Compared with the SS group, the high-dose QZF group shows scattered lymphocyte infiltration and partial catheter dilation and the acinar is uniformly arranged; acinar cells decreased compared with control. In the low-dose QZF group, focal infiltration of lymphocytes is observed which is similar to the SS group. Comparing the hydroxychloroquine group with the high-dose QZF group, the infiltration of lymphocyte in the high-dose QZF group was improved.

It is displayed in Figure 1(d); TUNEL-positive cells were increased in the SS model compared to the control. However, HCQ-treated and high- and medium-dose QZF-treated animals had an evident decreased number of TUNEL-positive cells compared to the SS group, implying that QZF may have a positive effect on SS mice by alleviating cell apoptosis; even the high-dose QZF exhibit better effect than the HCQ-treated group. The inflammatory cytokines IL-6 were predominantly expressed in submandibular gland tissue in the SS group. The high-dose QZF group and hydroxychloroquine group could decrease IL-6 expression in submandibular gland tissue compared with the SS group and attenuate lymphocyte infiltration in SS rats (Figures 1(c) and 1(e)). For IL-10, it is of much importance in Treg cell proliferation and maintaining body immune balance [39]. The results in the present study found that the expression of IL-10 in submandibular gland tissue increases after hydroxychloroquine and high-dose QZF treatment (Figure 1(f)). These results indicated the positive influence of QZF on SS rats and could attenuate pathogenesis in submandibular gland tissue.

### 3.2. Decreased IL-17 Expression in Submandibular Gland Tissue in the QZF-Treated Group

T cell-derived proinflammatory cytokine IL-17 is implicated in inflammatory diseases for its multiple functions. Its key role in inflammatory immune response has been proven by extensive studies and has pleiotropic effects on multiple cell populations. Local IL-17 production in the submandibular gland was examined by measuring IL-17 expression level. It is found that IL-17 levels were markedly elevated in SS rats (Figures 2(a) and 2(b)). Moreover, QZF can significantly decrease IL-17 production compared with SS rats (*P* < 0.001). Besides, mRNA level was downregulated in hydroxychloroquine and QZF-treated rats compared with SS (*P* < 0.001) (Figure 2(c)). In addition, mRNA was downregulated in high- and medium-dose QZF compared with hydroxychloroquine (*P* < 0.001).

### 3.3. Autophagy Was Enhanced in the QZF Treatment Group

Autophagy is a cellular process of self-eating and self-protection mechanism in cells; the purpose is to maintain cellular homeostasis by degrading damaged, denatured, and aging macromolecular substances and has reported the involvement in the pathogenesis of autoimmune diseases [40, 41]. Autophagy was demonstrated implication in a range of immune processes, including antigen presentation to the immune system, pathogen removal and clearance, the immune cells' survival, and inflammation [42]. Both autophagy LC3-II/LC3-I ratio and LC3-II expression in the submandibular gland were measured by WB and IHC, respectively. The mRNA expression level of the LC3-II/LC3-I ratio was determined by RT-qPCR. Our data indicate that hydroxychloroquine and high-dose QZF markedly promote LC3-II/LC3-I ratio elevation and LC3-II-positive immunostaining compared with SS (Figures 3(a)–3(c)) and no change difference was observed between hydroxychloroquine and high-dose QZF which indicated the comparable potential on autophagy (Figure 3(c)). Furthermore, the mRNA level of the LC3-II/LC3-I ratio exhibited in Figure 3(d) was markedly promoted in hydroxychloroquine and high-dose QZF compared with SS (*P* < 0.001).

### 3.4. QZF Attenuates Sjögren's Syndrome via Inhibiting PI3K/Akt/HIF-1*α*/VEGF Signaling Pathways

To investigate the engagement of signaling pathways in the QZF treating rat SS model, western blot analysis was conducted for protein expression. The expression of PI3K, AKT, HIF-1*α*, and VEGF was determined. Western blot analysis demonstrated that PI3K, AKT, HIF-1*α*, and VEGF protein is enhanced in the SS group versus control (*P* < 0.001) (Figure 4). The QZF treatment group could reverse this trend with comparable effect in contrast to hydroxychloroquine without change difference (*P* > 0.05) (Figures 4(b) and 4(c)). Particularly, compared with hydroxychloroquine, high-dose QZF exhibits better in inhibiting HIF-1*α* (*P* < 0.001) and VEGF (*P* < 0.01) protein expression (Figures 4(d) and 4(e)). PI3K and AKT were activated in SS; the phosphorylated p-PI3K and p-AKT production were elevated significantly in SS (*P* < 0.001) (Figures 4(b) and 4(c)). The findings above indicate the participation of PI3K, AKT, HIF-1*α*, and VEGF in QZF therapeutic effect on the rat SS model.

### 3.5. QZF Downregulate PI3K/Akt/HIF-1*α*/VEGF mRNA Level

Quantitative real-time PCR analysis was performed to further probe the signaling pathway engagement. The mRNA levels in the SS group are elevated in all genes compared with control (Figure 5). The PI3K/Akt/HIF-1*α*/VEGF signaling pathways were inhibited in the QZF treatment group by downregulating the gene expression of Pik3r1, Akt, HIF-1*α*, and VEGF; therefore, the transduction signal was descended. The HIF-1*α* gene expression was significantly downregulated in high-dose QZF in contrast to hydroxychloroquine (*P* < 0.01) (Figure 5(c)).

## 4. Discussion

In our study, initially, hydroxychloroquine, high-dose QZF, medium-dose QZF, and low-dose QZF were administrated to experimental mouse accordingly for consecutive 10 weeks. The HE staining experiment was conducted to check histology, and the results showed that the SS model had manifested pathological phenomena, which are highly infiltrated lymphocytes, atrophic glands, and the significantly reduced acinar in number. Then, in the submandibular gland tissue of rats in the HCQ-treated and high- and medium-dose QZF-treated group, these pathological phenomena were alleviated. We also used TUNEL staining to detect cell apoptosis in submandibular gland tissues, and the results proved that there are more apoptotic cells in the SS model group than that in control and that the HCQ-treated and high- and medium-dose QZF-treated group could reduce cell apoptosis. At the same time, the immunohistochemical experiment was conducted to clarify the expression of IL-6, IL-10, and IL-17 in rats' submandibular gland tissue. Served as cytokines, IL-6 and IL-17, it can be highly expressed in Sjögren's syndrome model rats, causing lymphocyte infiltration and inflammation. The expression of IL-17A is consistent with the results measured by immunohistochemistry. Th 17 cell produces IL-17 also termed as IL-17A, a proinflammatory cytokine, which has been proved in multiple evidences from many animal models and patients with pSS that IL-17 is intimately relevant to the pathogenesis of pSS and is critical for induction and persistence of chronic inflammation [22, 43, 44].

The experiment found that the HCQ-treated and high-dose QZF-treated group can reduce the expression level of IL-6 and IL-17. On the other hand, IL-10 participates in the proliferation of Treg cells and is related to its functional regulation, maintaining autoimmune balance. And the findings illustrated that its expression increased in the HCQ-treated and high-dose QZF-treated group. The above results have proven that QZF has a therapeutic effect in the Sjögren's syndrome rat model. Furthermore, the therapeutic effect in the high-dose QZF-treated group is even stronger than that in hydroxychloroquine.

Then, aiming at investigating the possible molecular mechanism of QZF on the treatment of Sjögren's syndrome in rats, we used WB analysis to detect expression of PI3K, pPI3K, AKT, pAKT, HIF-1*α*, VEGF, etc. The LC3-II/LC3-I ratio is a typical autophagy maker, whose expression in submandibular gland tissue was estimated. RT-qPCR technology was used to determine their mRNA transcription. The obtained results indicate that the effect of QZF in Sjögren's syndrome rats may be related to PI3K/Akt/HIF-1*α*/VEGF signaling pathways for the hydroxychloroquine and QZF can inhibit not only the PI3K, AKT, HIF-1*α*, and VEGF protein expression but also the phosphorylated PI3K and AKT protein P-PI3K and p-AKT. As reported before, the PI3K/Akt signaling pathway can mediate cell proliferation, differentiation, cell survival, etc., and abnormal expression of this pathway exists in autoimmune diseases [45]. Additionally, it can integrate signaling pathways from the cellular environment and ultimately regulate cell autophagy response [46]. At the same time, Kurebayashi et al. [47] and other studies have shown that the use of PI3K/mTOR inhibitors and the inhibition of Akt activity can affect the differentiation of Th17 cells from CD4+ T cells and thus decrease the secretion level of IL-17 cytokine. The results in the present study demonstrated that the PI3K/Akt signal pathway was activated in SS rats, QZF could inhibit the phosphorylated protein expression, and the PI3K/AKT signal transduction was descended. A critical transcription modulator, HIF-1*α* can regulate the tumor microenvironment whose high expression contributes to cells adapting to the hypoxic microenvironment and is regulated by the PI3K/Akt pathway [48]. The results showed the upregulation of HIF-1*α*/VEGF in SS after the PI3K/Akt signaling transduction was activated. Besides, the HIF-1*α* mainly regulates the number and function of various immune cells including regulatory T cells in the local tissue hypoxia response induced by inflammation [49, 50]. Therefore, exploring the submandibular gland autophagy based on the PI3K/Akt/HIF-1*α* signal cascade reaction would help clarify the pathogenesis of SS. The HIF-1*α* transcription increases under hypoxic conditions induced by chemical substances, which could activate various microenvironmental factors, thereby regulating cell apoptosis and autophagy [51]. In our study, the autophagy was significantly enhanced in the hydroxychloroquine and high-dose QZF group. These results indicate that QZF may mediate tissue autophagy via downregulating PI3K/AKT/HIF-1*α*/VEGF signaling pathways, thereby attenuating the inflammation, and facilitating cell tissue repair to treat SS. Moreover, the gene transcriptions of PI3K, AKT, HIF-1*α*, and VEGF were downregulated by QZF as well.

## 5. Conclusions

We have identified the therapeutic effect of QZF on the SS mouse model whose efficacy appears to be prior to hydroxychloroquine (40 mg·kg^−1^/d) in high-dose QZF (58 g·kg^−1^/d). The present study illustrated the inflammatory mechanism of PI3K/Akt/HIF-1*α*/VEGF in submandibular gland inflammation by demonstrating QZF treatment mediates PI3K/Akt/HIF-1*α*/VEGF expression in SS. Moreover, inhibition of PI3K/Akt/HIF-1*α*/VEGF can alleviate the focal infiltration of lymphocytes in the submandibular gland and decrease the secretion levels of inflammatory cytokines. Though, aside from PI3K/Akt/HIF-1*α*/VEGF activation, the transduction signal cascade between them was not identified. We provided a new insight on SS therapy; these observations found in the present study could contribute to designing a potential target-based therapeutic strategy to regulate submandibular gland inflammation in SS.

## Figures and Tables

**Figure 1:** Effects of QZF on SS rats. (a) The average water intake of rats from 11 weeks aged to 20 weeks aged in control, model, hydroxychloroquine, and three Chinese medicine treatment groups. (b) The diagram of the submandibular gland index of rats. Error bars represent SD, *n* = 3. ^∗∗∗^*P* < 0.001 for change difference versus the SS model. ^##^*P* < 0.01 and ^###^*P* < 0.001 QZF-treated group versus hydroxychloroquine. (c) HE staining of submandibular glands of rats. Red arrows indicate tissue infiltration. Scale bar = 50 *μ*m (magnification, ×400). The nucleus of submandibular gland tissue cells was stained blue by hematoxylin, while the cytoplasm was stained red by eosin. (d) Detection of cell apoptosis in the submandibular gland tissue of rats by TUNEL assay (scale bar = 50 *μ*m, magnification, ×400). The brown color represented the TUNEL-positive cells and blue, the nucleus pulposus. (e, f) Immunohistochemical detection of IL-6 and IL-10 expression in the submandibular gland tissue. Scale bar = 50 *μ*m (magnification, ×400). The positive immunostaining was colored in brown.

**Figure 2:** (a) IL-17A protein expression in submandibular gland tissue detected by western blot. (Left) Bands of IL-17A and beta-actin served as the internal control for protein semiquantification. (Right) The relative expression of IL-17A. ^∗∗∗^*P* < 0.001 for change difference versus SS model. ^###^*P* < 0.001 QZF-treated group versus hydroxychloroquine. (b) Immunohistochemistry was conducted to clarify the expression of IL-17 in submandibular gland tissue. Scale bar = 50 *μ*m (magnification, ×400). The positive immunostaining was colored in brown. (c) The relative mRNA expression level was determined by RT-qPCR analysis. Results of IL-17A mRNA level were displayed by histogram. Error bars represent SD, *n* = 3. The significance of each group compared with SS was calculated, ^∗∗∗^*P* < 0.001.

**Figure 3:** Autophagy marker LC3-II/LC3-I changes in submandibular gland tissue. Western blot detection of (a) bands and (c) relative quantification of LC3-II/LC3-I changes. (b) LC3-II production in submandibular gland via IHC. Scale bar = 50 *μ*m (magnification, ×400). The positive immunostaining was colored in brown. (d) LC3-II/LC3-I mRNA level in submandibular gland was quantified by RT-qPCR analysis. Error bars represent SD, *n* = 3. ^∗^*P* < 0.05, ^∗∗^*P* < 0.01, and ^∗∗∗^*P* < 0.001 for change difference compared to the SS model. ^#^*P* < 0.05 and ^###^*P* < 0.001 QZF-treated group versus hydroxychloroquine.

**Figure 4:** (a) The strip chart of protein expression in six groups detected by western blot. The expression of *β*-actin was serving as the internal reference to relatively quantify the protein expression by densitometry. (b–e) The column diagram of protein expression detected by western blot. (b) PI3K and phosphorylated PI3K; (c) AKT and phosphorylated AKT; (d) HIF-1*α* and (e) VEGF. Error bars represent SD, *n* = 3. Calculation of statistical significance was performed in each group compared with SS, ^∗∗^*P* < 0.01 and ^∗∗∗^*P* < 0.001. ^##^*P* < 0.01 and ^###^*P* < 0.001 QZF-treated group versus hydroxychloroquine.

**Figure 5:** The relative mRNA expression determined by RT-qPCR analysis. Error bars represent SD, *n* = 3 biological duplication. ^∗^*P* < 0.05, ^∗∗^*P* < 0.01, and ^∗∗∗^*P* < 0.001 difference is significant in each group compared with SS. ^#^*P* < 0.05, ^##^*P* < 0.01, and ^###^*P* < 0.001 QZF-treated group versus hydroxychloroquine.

**Table 1:** The primers for RT-qPCR.

Primers	Sequences
LC3-II-F	CAGCTCAATGCTAACCAAGCC
LC3-II-R	CTCGTACACTTCGGAGATGGG
Pik3r1(PI3K)-F	CGAGACGGCACTTTCCTTGT
Pik3r1(PI3K)-R	CGGTGGCAGTCTTGTTAATGAC
LC3-I-F	CACCCATCGCTGACATCTATGAAC
LC3-I-R	CGAAGGTTTCTTGGGAGGCGT
HIF-1*α*-F	AGATCAGCCAGCAAGTCCTTC
HIF-1*α*-R	GGGACTGTTAGGCTGGGAAA
IL-17A-F	TCAATGCGGAGGGAAAGCTG
IL-17A-R	CCACCAGCATCTTCTCGACC
Akt-F	GCCGCCTGATCAAGTTCTCC
Akt-R	GGCTTCTGGACTCGGCAATG
VEGF-F	ATGGATGTCTACCAGCGAAGCTACTG
VEGF-R	GGTTTGATCCGCATGATCTGCA
GAPDH-F	AGGTCGGTGTGAACGGATTTG
GAPDH-R	TGTAGACCATGTAGTTGAGGTCA

## Data Availability

The data generated and analyzed to support the findings of this study are available from the corresponding author upon reasonable request.
